# Efficacy and Safety of Hybrid Comprehensive Telerehabilitation (HCTR) for Cardiac Rehabilitation in Patients with Cardiovascular Disease: A Systematic Review and Meta-Analysis of Randomized Controlled Trials

**DOI:** 10.1155/2023/5147805

**Published:** 2023-08-09

**Authors:** Zheming Yang, Xiaodong Jia, Jiayin Li, Zhu Mei, Lin Yang, Chenghui Yan, Yaling Han

**Affiliations:** ^1^College of Medicine and Biological Information Engineering, Northeastern University, Shenyang, Liaoning 110167, China; ^2^State Key Laboratory of Frigid Zone Cardiovascular Diseases (SKLFZCD), Cardiovascular Research Institute and Department of Cardiology, General Hospital of Northern Theater Command, Shenyang 110016, China

## Abstract

**Backgrounds:**

Cardiovascular disease (CVD) is a serious condition that poses threats to patients' quality of life and life expectancy. Cardiac rehabilitation is a crucial treatment option that can improve outcomes for CVD patients. Hybrid comprehensive telerehabilitation (HCTR) is a relatively new approach. In the context of pandemics, HCTR can minimize the risk of cluster infections by reducing hospital visits while delivering effective rehabilitation care. This study is aimed at assessing the efficacy and safety of HCTR as a secondary prevention measure for CVD patients compared to usual rehabilitation care.

**Methods:**

We searched PubMed, Embase, The Web of Science, The Cochrane Library, and PsychINFO for all related studies up to January 20, 2023. Two reviewers independently screened the titles and abstracts of potentially eligible articles based on the predefined search criteria. Data were analyzed using a comprehensive meta-analysis software (RevMan5.3).

**Results:**

Eight trials, involving 1578 participants, were included. HCTR and usual rehabilitation care provide similar effects on readmission rates (odds ratio (OR) = 0.90 (95% CI 0.69-1.17), *P* = 0.43) and mortality (odds ratio (OR) = 1.06 (95% CI 0.72-1.57), *P* = 0.76). Effects on Short Form-36 Health Status Questionnaire (SF-36) score were also similar (SMD: 1.32 (95% CI-0.48-3.11), *P* = 0.15). Compared with usual rehabilitation care, HCTR can improve peak oxygen uptake (VO_2_ peak) (SMD: 0.99 (95% CI 0.23-1.74), *P* = 0.01) and 6-minute walking test (6MWT) (SMD: 10.02 (95% CI 5.44-14.60), *P* < 0.001) of patients.

**Conclusions:**

Our findings indicate that HCTR is as effective as traditional rehabilitation care in reducing readmission rates and mortality and improving quality of life in patients with CVD. However, HCTR offers the added advantage of improving VO_2_ peak and 6MWT, measurements of cardiorespiratory fitness and functional capacity, respectively. These results suggest that HCTR can be a safe and effective alternative to traditional rehabilitation care, offering numerous benefits for CVD patients. *Clinical Study Registration Number.* This trial is registered with NCT02523560 and NCT02796404.

## 1. Introduction

Cardiovascular disease (CVD) is a group of conditions affecting the heart and blood vessels, which can lead to heart attack, stroke, or other serious health complications. It is a leading cause of death and hospitalization globally, with an increasing prevalence due to aging populations, unhealthy lifestyles, and rising obesity rates [1–3]. Effective long-term management is essential for secondary prevention of CVD [4], which includes lifestyle modifications, medication therapy, cardiac rehabilitation (CR), cardiovascular implantable electronic devices for telemetry (CIED), and regular follow-up [5, 6].

Cardiac rehabilitation is an integral part of the secondary prevention strategy for patients with CVD. It is a comprehensive program that involves exercise training, risk factor education, psychological support, and lifestyle modifications. CR has been proven to enhance the prognosis and quality of life of CVD patients, but its efficacy largely depends on patient participation and adherence [7–9]. Unfortunately, a significant number of patients fail to adhere to CR, partly due to barriers such as lack of access to trained professionals and facilities, inadequate supervision and monitoring, transportation issues, and personal motivation. With the emergence of telemedicine technology, remote monitoring and telerehabilitation have become promising options to enhance CR compliance.

Telemedicine refers to the use of communication and information technologies to deliver healthcare services remotely, including diagnosis, consultation, treatment, and education. Remote cardiac rehabilitation (CR) training is a rare occurrence in telemedicine [10–13], but it has gained attention recently due to the COVID-19 pandemic and the need for social distancing measures. Virtual visits provide a new approach to remote CR, which can reduce unnecessary hospital visits and lower the risk of cluster infections compared to conventional rehabilitation care [14]. To meet this demand, the hybrid comprehensive telerehabilitation (HCTR) program has emerged.

The HCTR program is a new form of telemedicine that combines the use of information and communication technologies with telesupervised exercise training for patients with cardiovascular disease (CVD) [15, 16]. HCTR allows patients to receive rehabilitation services remotely while being closely monitored by healthcare professionals. The program includes various components of cardiac rehabilitation, including exercise training, risk factor education, psychological support, and lifestyle modifications, delivered through telecommunication technology. Patients are provided with remote monitoring devices, such as wearable sensors or smartwatches, to track their vital signs during exercise training sessions. Healthcare professionals then use this data to adjust the intensity and frequency of exercise training to suit each patient's needs. The program not only provides a convenient and personalized alternative to traditional inpatient and outpatient rehab but also reduces the risk of exposure to infection associated with conventional rehabilitation care. This approach can enhance the long-term management and outcomes of CVD patients, particularly during the COVID-19 pandemic and beyond.

The HCTR program has shown promising results in improving cardiac function and reducing hospitalization in patients with CVD, as demonstrated in recent randomized controlled trials [17]. However, some clinical trials have revealed no significant benefit from HCTR [18, 19]. To determine the efficacy and safety of HCTR among patients with CVD, we aimed to conduct a meta-analysis. The results of this analysis will provide important information to guide clinical practice and improve the long-term management of CVD patients.

## 2. Materials and Methods

### 2.1. Study Design

The purpose of this meta-analysis was to assess the efficacy and safety of the HCTR program for secondary prevention in patients with CVD. To identify eligible randomized controlled trials (RCTs) of combined telerehabilitation testing interventions, a comprehensive search was conducted in several databases, including PubMed, Embase, Web of Science, Cochrane Library, and PsycINFO. The search terms used included “telerehabilitation,” “remote rehabilitation,” “virtual rehabilitation,” “exercise therapy,” and “remedial exercise.” This rigorous search strategy is aimed at identifying all relevant studies that meet the inclusion criteria for the meta-analysis.

### 2.2. Study Inclusion Criteria

To ensure the quality and relevance of the studies included in this meta-analysis, we established specific inclusion and exclusion criteria. Eligible studies had to meet the following criteria: (1) data with extractable outcome measures; (2) randomized controlled trials; and (3) patients with cardiovascular disease who agreed to receive hybrid integrated telerehabilitation. Studies were excluded if they only involved telemonitoring without rehabilitation exercise supervision.

In this meta-analysis, the primary endpoints were mortality and readmission for CVD, which are critical outcomes for assessing the efficacy and safety of the HCTR program. By focusing on these key endpoints, we aimed to provide more reliable evidence to guide clinical practice and improve the long-term management of CVD patients.

### 2.3. Screen Process and Data Extraction

To ensure the quality and reliability of the studies included in this meta-analysis, a rigorous selection and assessment process was conducted. First, duplicate articles were removed from the EndNote (version X9) reference management software. Then, the titles and abstracts of the remaining studies were independently screened for eligibility by two reviewers (YZM, JXD), with no time or language restrictions. Any disagreements were resolved by a third reviewer (LJY). All studies deemed eligible were then reviewed in full text by two independent reviewers (YZM, JXD) using the same selection criteria. To ensure that all relevant studies were included in the analysis, a comprehensive search was also performed by examining the reference lists of previously published comments and key articles retrieved. Study characteristics, including author information, publication year, geographic location, study design, patient characteristics, and effect sizes, were extracted for each eligible study. The quality of included studies was assessed using Cochrane tools and grading of recommendations for randomized controlled trials.

### 2.4. Risk of Bias (Quality) Assessment

We used Cochrane's Risk of Bias tool to evaluate the quality and risk of bias in the studies included in our research [20]. This tool assesses five quality parameters of each study, such as randomization processes, deviations from intended interventions, missing outcome data, outcome measurement, and selection of reported results. Each parameter was evaluated using three to four questions to determine if the final score indicated low, high, or unclear risk of bias in the data. Overall, our research used rigorous methods to ensure the quality and validity of our findings.

### 2.5. Statistical Analysis

In this meta-analysis, we used odds ratios (OR) or hazard ratios with 95% confidence intervals (CI) to report dichotomized results for each comparison. The continuous results of adherence were expressed as standardized mean difference. In cases where mean differences and standard deviations (SD) of repeated measures were unavailable, we calculated the mean by subtracting the value after the intervention from the value before the intervention and using the largest standard deviation before and after the intervention as the standard deviation for each group. Heterogeneity was assessed using *I*^2^, and a random effects model was used when *I*^2^ > 30%, and a fixed effects model was used when *I*^2^ ≤ 30%. We used RevMan 5.3 (RevMan 2015) to combine the results, and Stata Corporation Version 15.0 was used for publication bias and sensitivity analysis.

## 3. Results

### 3.1. Study Characteristics and Quality Assessment

A comprehensive search was conducted, which yielded 1379 studies from five databases, and an additional 329 studies were identified from reference lists. After duplicates were removed and eligibility criteria were applied, 8 randomized controlled trials (RCTs) were included in this meta-analysis, which involved a total of 1578 participants with cardiovascular disease (CVD). Of these, 788 patients were randomized to receive HCTR (85.8% male; mean age 64.5 ± 8.5 years), and 790 received usual care (84.75% male; mean age 65.1 ± 13.5 years). The follow-up period ranged from 4 to 24 months (Table 1). The flow diagram of the study selection process is presented in Figure 1.

### 3.2. Risk of Bias of Included Studies

In our research, we conducted a risk of bias assessment for eight studies, and the results are displayed in Figures 2 and 3. These figures provide a detailed evaluation of each study's potential sources of bias and the corresponding risk of bias score. By conducting a thorough risk of bias assessment, we aimed to ensure the validity and reliability of our research findings. We used rigorous methods to evaluate the studies and to mitigate any potential biases that could have impacted the results. Overall, this helps to strengthen the overall quality of our research.

### 3.3. Meta-Analysis Results

#### 3.3.1. Readmission Rates

Three studies, comprising a total of 983 CVD patients, were included in the analysis of readmission rates. The results showed no significant difference in the rate of readmission for CVD between the HCTR group and usual care group (OR = 0.90 (95% CI 0.69–1.17), *I*^2^ = 0%, fixed-effect model, *P* = 0.43) (Figure 4).

#### 3.3.2. Mortality

Three studies, which involved a total of 1081 CVD patients, were included to evaluate the effect of HCTR on mortality. The results showed that the mortality rate in the HCTR group was not significantly different from that in the usual care group (OR = 1.06 (95% CI 0.72-1.57), *I*^2^ = 0%, fixed-effect model, *P* = 0.76) (Figure 5).

#### 3.3.3. Peak Oxygen Uptake (VO_2_ Peak)

Three studies involving a total of 1,092 patients with cardiovascular disease (CVD) investigated the impact of HCTR on VO_2_ peak, a measure of maximal oxygen uptake. The results indicated that HCTR significantly increased VO_2_ peak when compared to the usual care group, with a standardized mean difference (SMD) of 0.99 (95% CI 0.23-1.74), *I*^2^ = 0%, using a fixed-effect model, and *P* = 0.01 (as shown in Figure 6).

Overall, these findings suggest that HCTR may be an effective intervention for improving VO_2_ peak in patients with CVD.

#### 3.3.4. 6-Minute Walk Test (6MWT)

Four studies involving a total of 1176 patients with cardiovascular disease (CVD) examined the effect of HCTR on the 6-minute walk test (6MWT). The results showed that HCTR led to a significant improvement in 6MWT compared to the usual care group. The standardized mean difference (SMD) was 10.02 (95% confidence interval (CI): 5.44-14.60), with an *I*^2^ of 37%, indicating low to moderate heterogeneity. The fixed-effect model was used, and the *P* value was less than 0.001 (Figure 7).

Overall, these findings suggest that HCTR can lead to improvements in 6MWT in patients with CVD. These results are important as 6MWT is a widely used test to evaluate functional capacity and prognosis in patients with CVD. The absence of publication bias adds further credibility to the results. However, it is important to note that these findings should be interpreted with caution due to the limited number of studies and the potential for other sources of bias. Further research is needed to confirm these findings and explore the mechanisms underlying the observed improvements.

#### 3.3.5. SF-36 Score

Four studies involving a total of 1013 patients with cardiovascular disease (CVD) examined the effect of HCTR on the SF-36 score, a widely used questionnaire to evaluate health-related quality of life. The results showed that there was no statistical difference in the SF-36 score between the HCTR and usual care groups. The standardized mean difference (SMD) was 1.32 (95% confidence interval (CI): -0.48-3.11), *I*^2^ = 47%, indicating moderate heterogeneity. The fixed-effect model was used, and *P* = 0.15 (Figure 8).

While the results suggest that HCTR does not significantly impact the SF-36 score in patients with CVD, it is important to note that the studies were limited in number and there may be other factors that could affect the results. Further research is needed to better understand the potential benefits and limitations of HCTR on health-related quality of life in patients with CVD.

### 3.4. Sensitivity Analysis

The results of the sensitivity analysis demonstrate the robustness and reliability of the findings regarding the association between HCTR and readmission rates (Figure 9(a)) and mortality (Figure 9(b)). Specifically, the analysis revealed that the inclusion or exclusion of any particular study did not have a significant impact on the overall effect size. This suggests that the observed effect is not driven by a single study or a small subset of studies but rather reflects a consistent pattern across the literature as a whole. Therefore, the results can be considered stable and reliable and provide strong evidence for the relationship between HCTR and the outcomes of interest.

## 4. Discussion

Cardiovascular disease (CVD) is a leading cause of morbidity and mortality worldwide, often accompanied by impaired cardiac function and decreased physical condition in affected patients [21]. CVD can result in a decline in physical condition, which manifests as reduced endurance, strength, flexibility, and overall physical performance [22]. As CVD progresses, it gives rise to various symptoms including shortness of breath, fatigue, and limitations in physical activities. These symptoms stem from diminished cardiac function, compromised blood flow, and impaired oxygen delivery to the tissues [23]. Consequently, interventions targeting the improvement of cardiac function and physical condition are crucial for managing CVD.

Nonpharmacological interventions, such as cardiac rehabilitation, have been identified as a key strategy for the secondary prevention of CVD [24]. Cardiac rehabilitation programs typically is aimed at promoting healthy lifestyles and reducing the incidence of CVD risk factors, with the ultimate goal of improving survival outcomes for patients with CVD. These programs often include a variety of interventions, such as exercise training, nutritional counseling, and psychosocial support, and are tailored to meet the individual needs of patients [25]. By adopting a comprehensive, multidisciplinary approach to the management of CVD, cardiac rehabilitation programs have been shown to have a positive impact on a range of outcomes, including exercise capacity, quality of life, and mortality rates. As such, these programs represent an important avenue for improving the long-term prognosis of patients with CVD, and should be considered a key component of any comprehensive treatment plan for these individuals [26, 27].

Cardiac rehabilitation programs typically begin with exercise therapy, which has been shown to have a range of benefits for patients with cardiovascular disease (CVD). Specifically, exercise therapy can improve cardiopulmonary function, delay the progression of atherosclerosis, alleviate symptoms of myocardial ischemia, and reduce overall and cardiac mortality rates [28]. However, it is important for CVD patients to exercise under supervision, as it can be risky for them to do so independently [28, 29].

The COVID-19 pandemic has further complicated matters, as face-to-face counseling for many chronic disease patients, particularly those with CVD, has been limited [30]. These patients are at high risk for severe illness if infected with the virus, which can significantly increase the risk of death. Additionally, poor patient compliance with cardiac rehabilitation remains a persistent challenge, with studies suggesting that adherence rates are often suboptimal [31–33].

The emergence of HCTR has provided a potential solution to these issues. HCTR can provide effective monitoring of the physical training of CVD patients, thereby promoting long-term adherence to therapy and reducing the risk of viral transmission. This approach has been shown to be safe, effective, and widely accepted by CVD patients, making it a promising tool in the ongoing fight against cardiovascular disease [34, 35]. Exercise therapy remains a cornerstone of cardiac rehabilitation for patients with CVD. The use of HCTR has the potential to increase patient compliance with therapy and reduce the spread of COVID-19, making it a valuable addition to the treatment options available for these individuals [36].

This meta-analysis included 8 randomized controlled trials involving 1578 patients. Of these, 788 patients received HCTR (85.8% men; mean age 64.5 ± 8.5 years), and 790 patients received usual care (84.75% men; mean age 65.1 ± 13.5 years). Previous research has shown that readmission rates and mortality are significant challenges faced by CVD patients [5]. Therefore, the results of this study are important for evaluating the efficacy of HCTR in improving these outcomes. The results did not show a significant elevation in either outcome measure between the HCTR and usual care groups. Quality of life was assessed using the SF-36 score, and there was no significant difference between the two groups in this regard.

Our findings suggest that HCTR has a generally favorable safety profile. The trials analyzed did not report any significant adverse events directly linked to the HCTR intervention, such as increased mortality or readmission rates. It is important to note that while the current evidence suggests that HCTR is a safe approach for cardiac rehabilitation in patients with cardiovascular diseases, the safety of HCTR may vary depending on factors such as patient selection, prescribed exercise intensity, and adherence to appropriate monitoring programs. We stress the importance of personalized assessment and diligent monitoring of patients throughout the HCTR program. Moving forward, it is crucial for future research to continue investigating and monitoring safety outcomes to further enhance our understanding of potential risks associated with HCTR.

Although HCTR may not have a direct impact on readmission rates, mortality rates, or overall quality of life, our study reveals a substantial improvement in cardiopulmonary function associated with HCTR. Specifically, we observed a significant enhancement in VO_2_ peak and 6MWT when comparing HCTR to routine care. This result suggests that HCTR could serve as a viable alternative to routine care by effectively enhancing patients' cardiopulmonary function and exercise capacity throughout the rehabilitation process. These findings highlight the potential of HCTR to optimize the recovery journey and contribute to improved outcomes for individuals undergoing rehabilitation.

However, it should be noted that the benefits of HCTR for cardiac rehabilitation may be related to the duration of the rehabilitation plan. Some studies have shown that compared with the control group, short-term rehabilitation plans may not significantly improve the Cardiac output of CVD patients, while long-term plans may have a more significant effect [18, 37, 38]. Therefore, more research is needed to assess the potential clinical efficacy of HCTR interventions more accurately and comprehensively.

There are several limitations to this study, including the small sample size of the RCTs included in the meta-analysis. Ongoing studies may provide additional information about the efficacy of HCTR in treating CVD patients. Additionally, this study did not evaluate the rehabilitation of patients with conditions other than CVD, and differences in the methods of conduction and monitoring of HCTR may also have influenced the results.

These findings suggest that HCTR can effectively improve the cardiac rehabilitation of CVD patients. However, it is important to note that the small sample size of the included RCTs and the variability in the conduct and monitoring of HCTR may have influenced the results. Therefore, further studies with larger sample sizes and standardized protocols are needed to provide more accurate and comprehensive information on the potential clinical efficacy of HCTR for managing CVD patients.

## Figures and Tables

**Figure 1:** Flow chart of systematic review and meta-analysis, representing the number of articles screened, assessed, and included in meta-analysis.

**Figure 2:** Risk of bias summary.

**Figure 3:** Risk of bias graph.

**Figure 4:** Forest plot showing the effects of HCTR compared with usual care on readmission rates of CVD patients. Fixed-effects models were used.

**Figure 5:** Forest plot showing the effects of HCTR compared with usual care on mortality. Fixed-effects models were used.

**Figure 6:** Forest plot showing the effects of HCTR compared with usual care on VO_2_ peak. Fixed-effects models were used.

**Figure 7:** Forest plot showing the effects of HCTR compared with usual care on 6MWT. Fixed-effects models were used.

**Figure 8:** Forest plot showing the effects of HCTR compared with usual care on SF-36 score. Fixed-effects models were used.

**Figure 9:** The sensitivity analyses of the readmission rates (a) and mortality (b) by omitting each single study.

**Table 1:** Baseline characteristics included in 8 studies.

Author, year	Study design	Number of patients (control/intervention)	Follow-up (months)	Age (mean ± SD) (control/intervention)	Male (%) (control/intervention)	Disease	Outcome(s)
Tsai et al., 2022 [17]	RCT	81 (41/40)	6	73.3 ± 5.0/75.6 ± 6.0	70.7/67.5	HF	6MWD, LVEF, readmission rates
Piotrowicz et al., 2020 [18]	RCT	850 (425/425)	12-24	62.2/62.6	88.5/88.7	HF	6MWD, readmission rates, mortality, VO_2_ peak, Qol
Bravo-Escobar et al., 2017 [19]	RCT	28 (14/14)	4-6	55.64 ± 11.35/56.5 ± 6.01	100/100	Coronary artery disease or a valvular intervention	Exercise capacity, risk profile, Qol
Snoek et al., 2021 [37]	RCT	179 (90/89)	6-12	73.6 ± 5.5/72.4 ± 5.4	84/72	Coronary artery disease or a valvular intervention	Mortality, VO_2_ peak
Frederix et a., 2015 [38]	RCT	140 (70/70)	6	61 ± 9/61 ± 8	79/96	Coronary artery disease or a valvular intervention	VO_2_ peak, HR
Smolis-Bak et al., 2015 [39]	RCT	52 (26/26)	12-18	65.1 ± 8.2/60 ± 8.5	84.6/96.1	HF	6MWD,mortality, readmission rates, VO_2_ peak
Peng et al., 2018 [40]	RCT	98 (49/49)	4-6	60 ± 5.0/60 ± 5.0	59.2/57.2	HF	6MWD, LVEF, Qol, HR
Piotrowicz et al., 2010 [41]	RCT	152 (77/75)	4-6	56.4 ± 10.9/60.5 ± 8.8	85/95	HF	6MWD, VO_2_ peak, Qol

HF = heart failure; RCT= randomized controlled trial; 6MWD = 6-minute walking test; LVEF = left ventricular ejection fraction; VO_2_ peak = peak oxygen uptake; HR = resting heart rate; Qol = quality of life.

## Data Availability

The statistical and image data used to support the finding of this study are included within the article.

## Additional Points

*Clinical Study Registration Number*. This trial is registered with NCT02523560 and NCT02796404.
